The article "Prevalence and Correlation of Metabolic Syndrome in Patients with Bipolar Disorder in NGHA, Riyadh" was retracted in 2023. Reasons: unreliable results or conclusions; lack of ethics approval or compliance; concerns about the data; concerns about the peer review.

# Prevalence and Correlation of Metabolic Syndrome in Patients with Bipolar Disorder in NGHA, Riyadh

**DOI:** 10.1155/2022/5847175

**Published:** 2022-07-18

**Authors:** Asma Alanazi, Saud Alsadhan, Sultan Aldosari, Abdullah Alharbi, Mohammed Albawardi, Saud Alrabah, Haifa Alhawas, Maram Albalawi

**Affiliations:** ^1^Department of Basic Medical Sciences, College of Medicine, King Saud Bin Abdulaziz University for Health Sciences (KSAU-HS), Riyadh, Saudi Arabia; ^2^King Abdullah International Medical Research Centre (KAIMRC), Riyadh, Saudi Arabia; ^3^Department of Biostatistics and Bioinformatics, King Abdullah International Medical Research Centre, Riyadh, Saudi Arabia

## Abstract

**Background:**

Metabolic syndrome is considered dangerous, especially to patients that are diagnosed with a mental condition such as bipolar disorder, since these types of patients can be difficult to deal with. Metabolic syndrome can lead to multiple cardiovascular diseases, strokes, and diabetes. A careful approach is important when it comes to facing a complex condition such as this. This research will contribute to giving more information about the prevalence and statistics of metabolic syndrome in bipolar disorder patients at NGHA, Riyadh. No published study in literature has investigated the prevalence of metabolic syndrome in patients with bipolar disorder in NGHA, Riyadh.

**Methods:**

The study was conducted among 191 adult male (66) and female (125) patients at NGHA, Riyadh. The medical records were used for the assessment of metabolic syndrome and referrals by using a chart review for individuals. The main variables are metabolic syndrome and bipolar disorder. It was conducted on both males and females. Data was collected on data collection form and further analysis on relations was made by using SAS (Version 9.4). Chi-squared test and the Wilcoxon Two-sample test for two-level continuous variables. *P* ≤ 0.05 was determined to be the significance level.

**Results:**

Out of 191 patients, 130 were obese, 85 had diabetes, and 89 were hypertensive. Additionally, 50 (40%) females and 29 (43.9%) males had metabolic syndrome, a total of 79 (41.4%) out of 191.

**Conclusion:**

The findings of this study indicate that there is an elevated prevalence of metabolic syndrome in bipolar disorder patients in NGHA, Riyadh. Highlighting the potential danger that people may not be aware of.

## 1. Introduction

Bipolar disorder, which was known as manic depression, is a mental abnormality where a person has a major and a sudden change of mood, and it consists of emotional highs, mania, or hypomania, where a patient may feel energetic and may get over thrilled, and lows, depression, where a patient gets sad and helpless. This abrupt mood fluctuation alters the patient's cognitive capacity, appraisal, and sleep [1, 2]. Bipolar disorder is one of the chronic complicated psychological problems that have an early onset of presentation. Bipolar disorders are considered a range of disorders that include both bipolar I disorder and bipolar II disorder. Bipolar I disorder contains multiple phases of extreme mood episodes switching from depression to mania. However, bipolar II disorder is considered to be a milder form of mood raising that has a milder occurrence of hypomania which switches, with shifts, to extreme depression.

The article "Prevalence and Correlation of Metabolic Syndrome in Patients with Bipolar Disorder in NGHA, Riyadh" was retracted in 2023. Reasons: unreliable results or conclusions; lack of ethics approval or compliance; concerns about the data; concerns about the peer review.

Cyclothymic disorder explains short sessions of hypomanic symptoms which alternate with short sessions of depressive symptoms which are not as prolonged as seen in entire hypomanic sessions or entire depressive sessions [3]. A cross-sectional scanning of 11 countries indicated that bipolar disorders had a total lifetime prevalence of 2.4%, with 0.6% for bipolar type I and 0.4% for bipolar type II. The mean starting age of bipolar disorder is 25 years [4, 5]. Bipolar disorder is a disabling disorder that has a chronic course. 49 million people were suffering from bipolar disorder in 2013, which accounts for 9.9 million disability-adjusted life years (DALY) globally [6]. Additionally, patients that are diagnosed with any serious mental conditions, such as bipolar disorder and other mental illnesses, when compared to the general population, have higher rates of untreated medical conditions [7]. Unfortunately, they tend to die 10 to 30 years younger than other people, mainly due to cardiovascular diseases, stroke, and physical illnesses, which account for almost 60% of mortality [8].

A very common group of conditions that arise simultaneously, known as metabolic syndrome, can elevate the chances of type 2 diabetes, heart disease, and stroke. Conditions of metabolic syndrome include excess fat around the waist, increased blood sugar levels, elevated blood pressure, increased triglyceride levels, and decreased levels of HDL [9]. There are three main definitions for metabolic syndrome; we decided to work with the criteria of the International Diabetes Federation (IDF). Additionally, a reliable reporting of the aspects of metabolic syndrome can guide and provide the strategies for prevention and treatment [10]. Both bipolar disorder and metabolic syndrome are suggested to share similar predisposing factors, such as dysregulation of the sympathetic nervous system, endocrine disorders, and detrimental behaviors like smoking, overeating, use of alcohol, and lack of physical activity [4]. Moreover, psychotropic drugs that are used to treat bipolar disorder may result in weight gain and metabolic disruptions, including mutations in glucose and lipid metabolism. Additionally, metabolic syndrome increases the risk of developing cardiovascular diseases, consequently reducing a bipolar patient's life expectancy by 25 to 30 years. The precise mechanism of metabolic syndrome evolution in bipolar patients, however, is unclear. Other biological methods have been proposed, such as anomalies of the immune system, and disruption of the hypothalamic-pituitary-adrenocortical (HPA) axis. In the Middle East and North African region (MENA), a high prevalence of metabolic syndrome is noticed. In Tunisia, for example, it has been proclaimed to be 45.5% using the IDF criteria [11]. However, the prevalence of metabolic syndrome in bipolar disorder patients is rarely studied in Gulf Cooperation Countries (GCC). This research will contribute to giving more information about the prevalence and statistics of metabolic syndrome in patients with bipolar disorder in NGHA, Riyadh. No published study in literature has investigated the prevalence of metabolic syndrome in bipolar disorder patients in NGHA, Riyadh.

The article "Prevalence and Correlation of Metabolic Syndrome in Patients with Bipolar Disorder in NGHA, Riyadh" was retracted in 2023. Reasons: unreliable results or conclusions; lack of ethics approval or compliance; concerns about the data; concerns about the peer review.

## 2. Methods

### 2.1. Study Design, Area, and Setting

A retrospective cross-sectional study was conducted. The information was collected at one point in time; thus, a cross-sectional study is the best study design. The medical records were checked for the relationship between bipolar disorder and metabolic syndrome in adults. The study was conducted on bipolar disorder patients at King Abdulaziz Medical City in Riyadh, and the data was collected from the Ministry of National Guard Health Affairs NGHA. Established in May 1983, King Abdulaziz Medical City in Riyadh has a bedding capacity of 1501 beds. It provides all types of care to all National Guard soldiers and their families, beginning from primary health care, to complex tertiary specialized care.

### 2.2. Study Subjects

This study constitutes adult male and female bipolar patients older than 18 years. Bipolar patients are patients with a mental disorder that causes unexpected switches in energy, activity levels, mood, concentration, and the ability to carry out ordinary day-to-day tasks. Based on the availability of variables, the sample size was determined to be 191, 125 females and 66 males. A non-probability convenient sample was used. Patient records that met the inclusion criteria between March 2015 and December 2020 were included in the study.

### 2.3. Data Collection Process

All the information and data needed for this study were obtained by reviewing the medical records in the BESTCare system. This study was approved by the institutional Review Board (IRB) from King Abdullah International Medical Research Centre (KAIMRC) IRB #SP21R/247/05. The records were reviewed by the co-investigators. Metabolic syndrome was diagnosed based on the definition of the International Diabetes Federation (IDF).

The article "Prevalence and Correlation of Metabolic Syndrome in Patients with Bipolar Disorder in NGHA, Riyadh" was retracted in 2023. Reasons: unreliable results or conclusions; lack of ethics approval or compliance; concerns about the data; concerns about the peer review.

### 2.4. Data Analysis

The data was coded for entry and analysis using SAS (Version 9.4). For categorical variables, data are presented as frequency and percentage. We used the Chi-squared test and the Wilcoxon Two-sample test for two-level continuous variables. *P* ≤ 0.05 was determined to be the significance level.

## 3. Results

A total of 191 patients (125 females and 66 males) were included in the analysis. A retrospective chart review showed that the mean value for body mass index (BMI) for female patients was 33.76. Similarly, for male patients, it was 33.39, and when including all patients, it was 33.63. According to the IDF, both male patients' and female patients' mean values are considered obese. Furthermore, female patients had a higher prevalence of obesity. 89 (71.2%) female patients, and 41 (62.1%) male patients were obese, which is 130 (68.1%) out of 191 patients. The minimum value for BMI was 17.67, and the maximum value was 63.54.

The mean value for systolic blood pressure (SBP) for female patients was 128.42 compared to 131.44 for male patients. As for all patients, it was 129.47. According to the IDF, the mean SBP value for female patients is considered normal, whereas the mean value for male patients is elevated. Moreover, elevated SBP was observed to be found more in male patients than in females. 54 (43.2%) female patients and 35 (53%) male patients had elevated SBP, which is 89 (46.6%) out of 191 patients. The minimum value for SBP was 81, and the maximum value was 198.

The mean value for fasting blood sugar (FBS) for female patients was 6.68, and for male patients, it was 7.74. As for all patients, it was 7.04. Both male and female mean values are considered high according to the IDF. Additionally, 56 (51.9%) female patients and 29 (52.7%) male patients had elevated FBS, which is 85 (52.2%) out of 163 patients. The minimum value for FBS was 2.60, and the maximum was 40.30.

The mean value for high-density lipoprotein (HDL) levels for female patients was 1.22 and 0.97 for male patients. As for all patients, it was 1.14. It is important to mention that HDL is the only variable that leads to metabolic syndrome when reduced, rather than elevated as seen in all other variables. Although the IDF's benchmark is different for males and females, both mean values are considered to be reduced. Also, 68 (60.2%) female patients and 41 (67.2%) male patients had reduced HDL levels, which is 109 (62.6%) out of 174 patients. The minimum value for HDL was 0.54, and the maximum value was 2.16.

The article "Prevalence and Correlation of Metabolic Syndrome in Patients with Bipolar Disorder in NGHA, Riyadh" was retracted in 2023. Reasons: unreliable results or conclusions; lack of ethics approval or compliance; concerns about the data; concerns about the peer review.

The mean value for triglyceride levels was 1.38 for female patients and 1.86 for male patients. As for all patients, it was 1.55. In relevance to the IDF's definition, the mean value for females is considered normal, whereas the mean value for males is elevated. In addition to mean values, 25 (23.8%) female patients and 26 (44.1%) male patients had elevated triglyceride levels, which is 51 (31.1%) out of 164 patients. The minimum value for triglyceride was 0.25, and the maximum value was 5.25.

Even though these five variables are the diagnostic variables for metabolic syndrome according to the IDF, other non-diagnostic variables such as LDL and cholesterol levels are also considered important since they accompany HDL and triglyceride levels in the lipid profile test and, thus, they should be mentioned briefly. For cholesterol levels, the mean value for female patients was 4.55 and 4.64 in male patients. For LDL levels, the mean value for females was 2.82 and 2.98 in male patients. As for all patients, it was 4.58 for cholesterol and 2.88 for LDL. The minimum values for cholesterol and LDL were 2.15 and 0.84, whereas the maximum values were 9.02 and 6.92, respectively. For the mean value and prevalence of all variables, see Tables 1, 2, and 3.

When it comes to the prevalence of metabolic syndrome, 50 (40%) females and 29 (43.9%) males had metabolic syndrome, a total of 79 (41.4%) out of 191. When observing the mean values and percentages for all diagnostic variables, male patients were dominant in all except for BMI. Thus, male patients were expected to have a higher prevalence of metabolic syndrome even though obesity is the predominant variable in diagnosing metabolic syndrome according to the criteria of the IDF.

## 4. Discussion

In Saudi Arabia, this is the first study to assess metabolic syndrome in association with patients suffering from bipolar disorder. Only one research from Saudi Arabia assesses the prevalence of metabolic syndrome in patients with psychiatric disorders not bipolar disorder, however [12, 13]. Throughout the time of economic prosperity, Saudi Arabia's population's dietary patterns went through several alterations. According to some studies, obesity prevalence in adults spans from two-thirds to three-quarters of the population [4]. Women in this region have a higher prevalence of obesity than men; other studies have found. Additionally, metabolic syndrome is also more prevalent in women than in men in this region [14].

The prevalence of metabolic syndrome varies from 29.6% to 36.2% in males and 36.1% to 45.9% in females. The rates are comparable to those found in other Arab countries. Also, both diabetes mellitus and hypertension are prevalent [3, 15].

The article "Prevalence and Correlation of Metabolic Syndrome in Patients with Bipolar Disorder in NGHA, Riyadh" was retracted in 2023. Reasons: unreliable results or conclusions; lack of ethics approval or compliance; concerns about the data; concerns about the peer review.

Various aspects, such as a sedentary lifestyle, poor eating habits, and physical inactivity, contribute to the region's high prevalence of metabolic syndrome [16]. Furthermore, high economic status, insufficient education, and advanced aging are other factors that contribute to the region's high prevalence of metabolic syndrome [17–19]. Metabolic syndrome was found to be prevalent in 35.7% of bipolar patients in a Brazilian study [20]. This ratio, however, is comparable to that of the Brazilian general population. Metabolic syndrome is more prevalent in bipolar patients who take antipsychotic medications than in those who do not [21]. Metabolic syndrome is less common in patients who take a mood stabilizer only than in those who take an atypical antipsychotic or a polytherapy of an antipsychotic and a mood stabilizer. Patients with bipolar disorder who have metabolic syndrome have a poor prognosis, function, and insight, as well as recurrent hospitalizations, and a higher chance of developing tardive dyskinesia [22]. The region's high prevalence of metabolic syndrome in the general population can be partly responsible for the development of bipolar disorder.

Women in the region have a higher prevalence of metabolic syndrome and cardiovascular disorders, which could be a result of the region's torrid temperatures preventing people from performing outdoor activities in addition to the social norms. Nowadays, a large number of women work away from home do not have time to cook a proper healthy meal; as a result, an increasing number of families primarily rely on unhealthy junk food. Moreover, studies illustrated a genetic predisposition to diabetes in the Arabian population [23, 24].

A large number of bipolar patients live the majority of their lives depressed, denoted by anhedonia and poor energy, which may lead to a proclivity for an inactive lifestyle and metabolic syndrome. Treatment for bipolar disorder patients is not limited to psychological and pharmacological treatments, but also consists of lifestyle alterations, including, among other things, exercise, and healthy eating habits.

## 5. Limitations

This study had multiple limitations. To begin with, this study only included bipolar patients that were admitted to NGHA, Riyadh. Additionally, the cross-sectional design limited access to the patients' data, since all the information and data needed for this study were obtained by reviewing the medical records from the electronic health record database BESTCare. Furthermore, some patients were missing some variables. Out of 191 patients, 28 patients (17 female and 11 male) were missing FBS, 17 patients (12 female and 5 male) were missing HDL, 27 patients (20 female and 7 male) were missing triglyceride, 16 patients (12 female and 4 male) were missing cholesterol, and 17 patients (12 female and 5 male) were missing LDL. As for blood pressure to assess hypertension, we only worked with SBP since all patients had its readings, whereas 108 patients (58 female and 40 male) were missing DBP (diastolic blood pressure) readings (56.5%).

The article "Prevalence and Correlation of Metabolic Syndrome in Patients with Bipolar Disorder in NGHA, Riyadh" was retracted in 2023. Reasons: unreliable results or conclusions; lack of ethics approval or compliance; concerns about the data; concerns about the peer review.

## 6. Conclusion

Metabolic syndrome is a serious hazard to patients with bipolar disorder since it leads to a poor prognosis and poor quality of life (QOL). A thorough and careful approach is required to confront this rising issue with high urgency, in order to achieve greater control of the disorder.

## Figures and Tables

**Table 1:** Mean, minimum, and maximum values for all patients (*n* = 191).

Variables	Mean ± SD	Minimum	Maximum
BMI	33.63 ± 7.64	17.67	63.54
Systolic BP	129.47 ± 23.93	81	198
FBS	7.04 ± 4.22	2.60	40.30
HDL	1.14 ± 0.29	0.54	2.16
Triglyceride	1.55 ± 0.93	0.25	5.25
Cholesterol	4.58 ± 1.11	2.15	9.02
LDL	2.88 ± 1.00	0.84	6.92

**Table 2:** Mean, minimum, and maximum values with a comparison between male and female patients (n Males =66) (n Females =125).

Variables	Mean ± SD (males)	Mean ± SD (females)	Minimum (males)	Maximum (males)	Minimum (females)	Maximum (females)
BMI	33.39 ± 8.15	33.76 ± 7.39	19.72	63.54	17.67	51.08
Systolic BP	131.44 ± 21.07	128.42 ± 25.34	84	193	81	198
FBS	7.74 ± 5.73	6.68 ± 3.17	2.60	40.30	4.10	21.10
HDL	0.97 ± 0.24	1.22 ± 0.28	0.54	1.69	0.67	2.16
Triglyceride	1.86 ± 1.02	1.38 ± 0.83	0.72	5.25	0.25	5.15
Cholesterol	4.64 ± 1.31	4.55 ± 0.99	2.53	9.02	2.15	7.00
LDL	2.98 ± 1.18	2.82 ± 0.89	0.84	6.92	0.90	4.88

**Table 3:** Prevalence of metabolic syndrome and its associated signs and symptoms with a comparison between male and female patients.

Variables	*n* (Males)	%	*n* (Females)	%	*n* (Total)	%
Elevated BMI	41	62.1% (Males) 21.47% (Total)	89	71.2% (Females) 46.60% (Total)	130	68.06%
Elevated SBP	35	53.03% (Males) 18.32% (Total)	54	43.2% (Females) 28.27% (Total)	89	46.59%
Elevated FBS	29	52.73% (Males) 17.79% (Total)	56	51.85% (Females) 34.36% (Total)	85	52.15%
Reduced HDL	41	67.21% (Males) 23.56% (Total)	68	60.18% (Females) 39.08% (Total)	109	62.64%
Elevated triglycerides	26	44.07% (Males) 15.83% (Total)	25	23.81% (Females) 15.24% (Total)	51	31.07%
Metabolic syndrome	29	43.9% (Males) 15.18% (Total)	50	40% (Females) 26.18% (Total)	79	41.36%

## Data Availability

The authors confirm that the data supporting the findings of this study are available within the article and its supplementary material.
